# The Application of the Unsupervised Migration Method Based on Deep Learning Model in the Marketing Oriented Allocation of High Level Accounting Talents

**DOI:** 10.1155/2022/5653942

**Published:** 2022-06-06

**Authors:** MengYang Liu, MingJun Li, XiaoYang Zhang

**Affiliations:** ^1^Department of Financial Assets, Shandong Labor Vocational and Technical College, Jinan 250000, Shandong, China; ^2^Department of Labor Economics, Shandong Labor Vocational and Technical College, Jinan 250000, Shandong, China; ^3^College of Humanities, Shandong Agriculture and Engineering University, Jinan 250000, Shandong, China

## Abstract

Deep learning is a branch of machine learning that uses neural networks to mimic the behaviour of the human brain. Various types of models are used in deep learning technology. This article will look at two important models and especially concentrate on unsupervised learning methodology. The two important models are as follows: the supervised and unsupervised models. The main difference is the method of training that they undergo. Supervised models are provided with training on a particular dataset and its outcome. In the case of unsupervised models, only input data is given, and there is no set outcome from which they can learn. The predicting/forecasting column is not present in an unsupervised model, unlike in the supervised model. Supervised models use regression to predict continuous quantities and classification to predict discrete class labels; unsupervised models use clustering to group similar models and association learning to find associations between items. Unsupervised migration is a combination of the unsupervised learning method and migration. In unsupervised learning, there is no need to supervise the models. Migration is an effective tool in processing and imaging data. Unsupervised learning allows the model to work independently to discover patterns and information that were previously undetected. It mainly works on unlabeled data. Unsupervised learning can achieve more complex processing tasks when compared to supervised learning. The unsupervised learning method is more unpredictable when compared with other types of learning methods. Some of the popular unsupervised learning algorithms include k-means clustering, hierarchal clustering, Apriori algorithm, clustering, anomaly detection, association mining, neural networks, etc. In this research article, we implement this particular deep learning model in the marketing oriented asset allocation of high level accounting talents. When the proposed unsupervised migration algorithm was compared to the existing Fractional Hausdorff Grey Model, it was discovered that the proposed system provided 99.12% accuracy by the high level accounting talented candidate in market-oriented asset allocation.

## 1. Introduction

Deep neural networks and machine learning have been overlooked by the investment management industry because of their phenomenal progress and current state of the art in several fields, such as natural language understanding, computer vision, and speech recognition [1]. Deep neural networks and machine learning have been overlooked by the investment management industry because of their phenomenal progress and current state of the art in several fields, such as natural language understanding, computer vision, and speech recognition. Inadequate data in the banking sector is just one of the elements that has led to this predicament [2]. Due to a lack of training data, poor generalisation in out-of-sample data, and an intrinsically low signal-to-noise ratio in financial time-series data, deep learning algorithms have been unable to outperform conventional approaches. A very large number of hand-crafted indicators is required in order to attain the absolute bare minimum. If the predictive ability of one indicator reduces over time, it may be essential to construct a new indicator to compensate [3]. Deep learning models have the ability to learn new features after being exposed to a large amount of additional data. If desired, these weights can be determined by policy rather than model parameters, allowing for greater flexibility. To achieve walk-forward learning in deep neural network models, hyperparameters, which impact how quickly the model responds to new data, must be carefully chosen, as described above. Point estimates of anticipated returns are frequently found to be wrong in financial time-series data due to the low signal-to-noise ratio of the underlying data [4]. This makes it necessary to employ a Bayesian framework in your financial decisions, which takes into account both projected returns and estimates of uncertainty. Establish new training objectives for accounting employees by identifying market requirements, deconstructing the accounting major into its constituent elements, and then constructing the accounting major again [5]. Combining classroom practice training with accounting personnel quality training, accounting personnel quality training, and accounting personnel quality training results in an improvement in the overall quality of students [6]. The upshot is that China has coined the term “big data,” which refers to the fact that data is collected and organized into a well-organized database and that specialists are being trained to manage data quality and increase its availability as a result of these advancements in the country. Due to the high cost of labor in China, the time and effort required to teach management accounting skills using big data technologies to workers is prohibitively expensive [7].

Accounting relies on the organization to provide them with correct and dependable information in order for them to function properly. Structured data and unstructured data are the two most fundamental sorts of information to understand [8]. Trade secrets must be protected while providing investors with an unstructured accounting report while also withholding some information from them. A trade secret protection balance must be struck between providing investors with an unstructured accounting report and also withholding some information from them [9]. In an environment where all parties have equal access to the same information, it becomes easier for each organization to communicate with its consumers and suppliers, hence reducing competition. In recent years, the increased availability of data information has made it easier for investors to make better investment decisions, which has benefited both investors and financial markets. As a result of the increasing transparency and clarity in this approach to investing in recent years, investors have developed an increased trust in asset pricing and cost-benefit analyses [10]. Traditional payment reimbursement and the processing of even the most basic data have witnessed a dramatic drop in recent years as a result of improved transparency and data sharing across the board. Because of the increasing demands of the big data age, accounting professionals must reevaluate their skills and abilities to keep up with the pace of change. Meanwhile, financial reimbursements are being reduced [11]. The platform will provide government agencies with more specific corporate data information in order to aid them in better managing and using the company's data. However, the vast majority of data that is used by the federal government is collected through the data sharing procedure. To provide continuous financial auditing and advisory services to clients, data from the platform must be made available to the company's internal management and internal audit control departments. To ensure that their organizations' financial earnings are maximised, accountants must be constantly adapting their practices to the ever-changing nature of the business world. Honesty and integrity are two of the most important characteristics in accounting [12]. In order to keep up with the rapid rate of innovation and advancement that will benefit all of society, it is vital that accountants' learning capacities be improved. To remain relevant in today's culture, accountants must constantly acquire and master new skills and practices. This requires them to stay on top of the latest technological advances. Aside from that, accountants must be able to communicate and engage with their coworkers in an appropriate and professional manner.

Businesses and other sectors of society are becoming increasingly reliant on management accountants to provide financial reporting and analysis to their stakeholders [13]. It is essential to have a supportive social and organizational environment in place in order to properly manage accounting talent and achieve success. It is necessary for all units of society to strictly implement the training requirements for accountants before implementing any training requirements for accounting professionals in order to ensure that accountants learn from practical actions and to increase the number of opportunities for accounting professionals to train accountants from practical actions [14]. It is critical for organizations to identify and specify the requirement for accounting personnel training as soon as possible. If educational institutions want to meet the needs of workers in the big data business, they must adapt their curriculum settings as soon as feasible, and educational resources must be incorporated into their programmes [15]. By viewing this video, you will learn how to improve your accounting abilities. For an enterprise accounting professor to fully grasp how big data affects workforces, he or she must connect government policy to accounting talent development trends and design an online platform to train accountants in accordance with the specific requirements of this organization [16]. Having a robust self-management system in place is crucial for the success of any organization. It is vital to build an effective talent evaluation system and to improve the management of talent assessment in order to identify competent management accountants for training on campus or through social media. In turn, they are able to provide short-term intensive training and evaluation, boost liquidity among appropriate accountants, and minimise the rigidity of the accounting sector within the organization [17]. As a result of the growth of new media, there has been a substantial shift in the rate at which information is disseminated as well as the impact that information has on society as a whole in the information age. Accountants who want to advance and succeed in this new era of accounting ethics must keep up with the latest developments and understand socialist principles, which are becoming increasingly common in the profession [18]. Spreading the spirit and principles of this new age through various media channels would encourage everyone to take responsibility for their own societal obligations, while also improving the general mood of the general public, which would be beneficial. In the face of constantly changing legislation, being able to rely on an independent audit department ensures that audit work is authoritative and impartial in nature [19]. The employment of auditing responsibilities by organizations can help them to ensure that they are operating in a fair and impartial manner, as well as monitor and analyze the financial practices of the organization [20].

Motivate and educate all members of the accounting team on the importance of adhering to and understanding all applicable laws and ethical standards, as well as the organization's responsibilities to the broader public sector community and other stakeholders [21]. If you are doing both types of investigations at the same time, it is not suggested that you perform internal and external audits simultaneously. The release of audit findings provides an additional motivation for accountants to perform their jobs well [22]. You should take into consideration the advantages of training and appraising your accounting staff. The establishment of an ethics code for accountants is a never-ending process that will be completed eventually. In order to keep on top of the quickly changing environment in which they work, accountants must develop new concepts and procedures, as well as chart a course toward greater social responsibility [23]. A person who wants to extend their views and be open to new possibilities in their life needs to have the self-discipline of an accountant to do so. Upon completion of a thorough examination of their practices, accounting departments are obligated to document their ethics and social responsibility in the company's archives [24]. As a result of the requirement for a talent team to aid in the management of big data organizations, the formation of a talent pool becomes important when it comes to accounting for big data as well as when it comes to financial big data management. Large amounts of accounting data can be comprehended in terms of both size and volume of data, which allows for the formation of a new type of work team and the transformation of the accounting management work mode [25]. However, even while we may continue to rely on our accounting management team, we must support them in their attempts to change the old accounting management work pattern. The study proposed AI based novel approach for liver screening and prediction by using convolution neural network [26]. The performance of the image fusion process can also be improved with a new deep belief network-based framework [27]. It is also possible to find the best values for the hyperchaotic map's parameters and encryption factors by using a multiobjective optimization technique. Selecting the best features from medical images can be done using multiobjective differential evolution. Then, the coefficient of determination and the energy loss-based fusion functions are used to obtain the fused coefficients [28]. Using an intruder to seize a few nodes, a node capture attack is used to gain control of the entire WSN by obtaining the WSN's useful information, such as keys, routing mechanisms, and data. The study proposed a Black Hole Optimization Algorithm (BHOA) on the best possible node capture attack in order to discover the optimal nodes with the best chance of attack in WSNs [29]. This study focused on marketing oriented asset allocation of high level accounting talents using unsupervised migration method based on deep learning.

## 2. Proposed Method

Asset allocation is a strategy for balancing risk and returns by investing in different asset classes. The historical price movements of other asset classes like equity, fixed income or debt, or gold are analyzed. The low or negative correlation among these asset classes is taken into account. Hence, diversification across asset classes can considerably reduce the risk and generate significant returns in the long term. Financial experts suggest that the right asset allocation strategy is crucial to achieving your financial goals. Accountants at higher levels are involved in formulating company budgets and developing economic models. In addition to this, accountants prepare and file taxes for the company. After the final analysis, they will recommend reducing total tax liabilities in the future. Machine learning (ML) is applied in the marketing oriented asset allocation of high level accounting talents. In this study, the advantages and disadvantages of applications of unsupervised migration are analyzed. The process of high level accounting talent with the support of artificial intelligence is given in Figure 1. The main advantage of implementing an unsupervised machine learning algorithm includes clustering: It automatically categorizes the dataset based on their similarities. Anomaly detection discovers unusual data points in the dataset; with the help of it, fraudulent transactions are detected. Association mining identifies groups of items that appear frequently together in a given dataset. Latent variable models are widely used in data preprocessing need to supervise the model; it helps to find all kinds of unknown patterns in the data. However, this model has certain drawbacks too, and they are that there is no precise information regarding data sorting and less accurate results. The user needs to spend more time interpreting and labelling the classes.

The role of Artificial Intelligence in Figure 1 is as follows.

1. Fraudulent Transaction Detection: AI has programmed fraud detection. It prevents fraudulent actions by analyzing patterns and monitoring every document in the company. AI checks the accounts as per accounting rules and laws. AI takes the issue to accountant for second check.
2. Automation of Data Input: AI can read, analyze, and process all the documentation without any flaw. It reduces human effort in data input.
3. Indicating Due Date: The AI indicates the due dates and raises invoice for each contractor.
4. Forecasting and Auditing: The machine learning algorithms create good view in forecasting. Auditing task is also carried out by the AI itself. Auditing is an important process in accounting. AI audits with high accuracy and efficiency.
5. Risk Management: AI prevents risk by identifying it. The quick access of AI to all data's and predicting models is more beneficial in this case.
6. Closing Procedure: AI can support the accountant or even carry out tasks automatically without the intervention of humans in monthly or quarterly closing procedures.
7. Hidden Details: AI is capable of discovering hidden patterns and trends, thus helping the company.

Thus, computers using AI in accounting have proven to be great in performance when compared to humans. It carries out tasks of deep insight and also handles repetitive and time-consuming tasks at ease. The time consumed by human fatigue and human error in accounting is totally avoided. Therefore, it gives more time for other tasks to the accountants who handle them. In this research, candidates with high level accounting talents are expected to have good knowledge of market-oriented asset allocation. The performance of these candidates through an unsupervised learning mechanism is considered with the aid of an intelligent networking system.

### 2.1. Unsupervised Migration Algorithm

Marketing oriented asset allocation of high level accounting talent research decisions is typically based on classification techniques used to categorize a set of measurements. Various data classification methods are used to determine an organization's overall marketing oriented asset allocation of high level accounting talents crisis using historical data. It is critical to identify suitable parameters (features) that are critical for the development of an accurate marketing oriented asset allocation of high level accounting talent crisis prediction unsupervised migration algorithm. This is known as an “attribute selection problem,” and it helps improve the classifier's performance.

The proposed unsupervised migration algorithm has been split into two categories: unsupervised feature extraction and migration algorithm-based data preprocessing. Within that suggested work, the implementation of the unsupervised migration algorithm with information to identify and categorize process includes some of the following processes. The unsupervised migration algorithm performs feature extraction and chooses the appropriate set of attributes.

Instead, the selected feature subset is applied to the classification stage using WEN and AI techniques. In this manner, the unsupervised migration algorithm with deep learning categorizes marketing (online or offline) oriented asset allocation of high level accounting talents data and predicts whether an organization will experience a marketing (online/offline) oriented asset allocation of high level accounting talents crisis.

As a result, the statistical analysis that occurs in the *M*_*i*_^*k*^(*h*) high level accounting talents solution has been acknowledged, and each statistical analysis for the balanced depending on the number of times it appears in the |*τ*_*i*_(*h*)^*∞*^|.|*i*|^*β*^ marketing assets has been acknowledged. A higher *i* value is assigned to the characteristics that appear more frequently within the set of best approaches. If a feature is enabled in all of the ∑_*nϵj*_*k*__|*τ*_*n*_(*s*=*h*)^*∞*^|.|*ŋ*_*n*_|^*β*^ best approaches, then *nϵl*_*k*_. If, on the other hand, a feature is not enabled at all, *i* = 0. Using the probability *L*_*i*_^*p*^(*s*), a novel hybrid algorithm with feature *j* determines whether or not feature *i* is chosen (*s*) following the equation

(1) $$\begin{array}{c} M_{i}^{k}\left(h\right)=\overset{j=1}{\underset{i=0}{\sum }}\left\{\begin{array}{cc} \frac{\left|\tau_{i}{\left(h\right)}^{\infty }\right|.{\left|i\right|}^{\beta }}{\sum_{n\epsilon j_{k}}\left|\tau_{n}{\left(s=h\right)}^{\infty }\right|.{\left|{ŋ}_{n}\right|}^{\beta }} & \mathrm{if}\;n\epsilon l_{k}\\ 0 & \text{otherwise} \end{array}\right.. \end{array}$$

In this equation *l*_*k* _ is the number of parameters which can be included with the short-term solution; *τ*_*i*_ and *τ*_*n*_ are the analysis value but also methodology desirability of the functionality The parameters *τ*_*i*_ regulate the market merits of the asset allocation of high level accounting talents statistical analysis used to the migration algorithm.

Whenever the whole migration algorithm did find their own first solution for the marketing asset allocation of high level accounting talents, the analysis elimination among all modules begins, but every insect *k* invests the amount of training and testing statistical analysis given by the following equation

(2) $$\begin{array}{c} \tau_{i}^{k}\left(h\right)=\sum_{i=1}^{j=0}\left\{\begin{array}{cc} \emptyset .\gamma \left(E^{k}\left(h\right)\right)+\int \frac{\emptyset \left(u-1E^{k}\left(h\right)i\right)}{r}, & \mathrm{if}\;i\in E^{k}\left(h\right)\\ 0 & \text{otherwise} \end{array}.\right. \end{array}$$

*h* (*u*)*k* is the highlight subset of online and offline marketing assets produced by ant *k* iteration and | *h*^*u*^ | *u* measures the time, and Δ is the parameter that controls the relative importance of feature subset length and ranges between 0 and 1. Equations (3) and (4) do the above processes.

(3) $$\begin{array}{c} \tau_{i}\left(h+1\right)=\sum_{i=1}^{g}\left(1-\rho 1\right)\tau_{i}\left(g\right)+\sum_{i=1}^{h}\Delta_{i}^{k}\left(h\right)+\Delta \tau_{i}^{n}\left(h\right). \end{array}$$

Whichever values are less than the prespecified value may be included in the guideline, which is referred to as the minimum and maximum level of statistical analysis for the marketing assets instances for each. Once the ants have exploited all of the attributes, the regulation process will be terminated. To generate standards, the ants employ a probabilistic model *M*_*ij*_, as shown in equation (5), from which they can select a parameter value.

(4) $$\begin{array}{c} M_{ij}=\frac{\Delta_{i}^{k}\left(h\right)+\Delta \tau_{i}^{n}\left(h\right)}{\sum_{i=1}^{d}\left(H_{i}\right).\sum_{j=1}^{n}\left(\Delta_{i}^{k}.\Delta \tau_{i}^{n}\left(h\right)\right)}. \end{array}$$

For each term *ij* that can be introduced to the current rule, the ant colony optimization method specifies the amount *ij* of an optimizer that represents the performance of this time frame in terms of its ability to improve the rule's predictive performance. The significance of *ij* for time frame *ij* is a measure of an electron density associated with that time frame. The result is approximated for each time frame *ij* as shown in equation (6).

The migration method specifies the amount *ij* of an optimization technique that signifies the performance of such a given timeframe in terms of the ability to enhance the prediction accuracy for each term *ij* which can be initiated to the current scheme. The importance of *ij* in terms of time frame *ij* denotes the electronic structure associated with just that time frame. As shown in equation (6), the result is estimated for each specified timeline *ij*.

(5) $$\begin{array}{c} E\left(ME_{i}=H_{ij}\right)=-\sum_{n=1}^{k}\left(M\left(E|E_{i}=H_{ij}\right).\;\log_{2}\sum M\left(n|E_{i}=\;H_{ij}\right)\right). \end{array}$$

It improves the minimum and maximum statistical report simplicity because a shorter training and testing regulation is easier to understand than a longer one. The statistical report is replanting process that begins once the ants have completed the marketing process. This method eliminates unnecessary reconstructed by ants at each step; thus, for improving rule quality, the asset value is enough according to equation (7).

(6) $$\begin{array}{c} H_{ij}=\int \frac{M\left(E|E_{i}=H_{ij}\right)}{\sum_{i=1}^{d}\left(H_{i}\right).\sum_{j=1}^{n}\left(\Delta_{i}^{k}.\Delta \tau_{i}^{n}\left(h\right)\right)}*\frac{M\left(n|E_{i}=\;H_{ij}\right)}{\sum_{i=1}^{d}\left(H_{i}\right).\sum_{j=1}^{n}\left(\Delta_{i}^{k}.\Delta \tau_{i}^{n}\left(h\right)\right)}. \end{array}$$

The marketing asset allocation of high level accounting talents uses this method to discover simplified as well as stronger classification training and testing. Initially, those online and offline are administered with the same quantity of analysis as specified in the following equation:

(7) $$\begin{array}{c} \tau_{ij}\left(h=0\right)=\int_{i=1}^{n}\frac{1}{\sum_{i=1}^{u}h=n_{i}}. \end{array}$$

The (WSN) nodes which were used by the current statistical report would be updated as the artificial intelligence transactions substance throughout all path investigation. It is necessary to simulate analysis evaporation at the same time. As a result, the recursive operative is executed in accordance with the following equation:

(8) $$\begin{array}{c} \tau_{ij}\left(h\right)=\int_{i=1}^{j}\left(1-\rho \right)\tau_{ij}\left(h-1\right)+\sum_{i=1}^{n}\left(1-\frac{1}{1+M}\right)\tau_{ij}\left(h-1\right). \end{array}$$

As such, in the statistical analysis rate of evaporation, *E* is the attribute as defined in equation (7), and *t* is the unique identifier of the iterative process training and testing. Endpoints that have not yet been used by current marketing oriented asset allocation on either will only have online and offline marketing assets analysis evaporation, as shown in the following equation:

(9) $$\begin{array}{c} \tau_{ij}\left(h\right)=\frac{\tau_{ij}\left(h-1\right)}{\sum_{i=1}^{d}\sum_{j=1}^{n_{i}}\tau_{ij}\left(h-1\right)}+\frac{M\left(n|E_{i}=\;H_{ij}\right)*M\left(E|E_{i}=H_{ij}\right)}{\sum_{i=1}^{d}\left(H_{i}\right).\sum_{j=1}^{n}\left(\Delta_{i}^{k}.\Delta \tau_{i}^{n}\left(h\right)\right)}, \end{array}$$

(10) $$\begin{array}{c} E\left(ME_{i}=H_{ij}\right)=\sum_{i=1}^{j=1}\frac{M}{E}\times H_{i}^{\#}+\frac{M}{E}\times H_{i}^{*}+\int \left(\frac{E}{2}+k_{j}\right)\times h\times Q^{\#}+\int \left(\frac{E}{2}+k_{j}\right)\times h\times E^{*}. \end{array}$$

In equation (11) different versions in marketing oriented asset allocation delivery times have a significant effect on various stages of protection systems required by distributors using the following equation:

(11) $$\begin{array}{c} k_{j}=\overset{j=1}{\underset{i=1}{\sum }}\sqrt{2\times M^{2}\times \int \frac{\sum H\times E\times M\times h\times \sqrt{2\pi r}}{\sum M\times H_{ij}}}. \end{array}$$

To make the equation clearer, the statistical power of exchange utilization is denoted by *M*, and the expense of not possessing inventory assets is denoted by *H*_*ij*_ in the following equation:

(12) $$\begin{array}{c} h_{ij}=\sum_{i=1}^{j}M_{i}\times \sum_{i=1}^{j}{\left(k_{i}+k\right)}^{2}. \end{array}$$

Marketing oriented asset allocation of high level accounting talents is used to collect data from large-scale quality management practices for the statistical analysis report, which is part of the training and testing process. The analytical network (AI and WSN) process is used to analyze the performance evaluation establishment of marketing oriented assets, and an enterprise marketing evaluation high level accounting is established in the following equation:

(13) $$\begin{array}{c} HM_{ij}=\sum_{i=0}^{j=1}\int \sqrt{k}=\sqrt{\sum_{i=1}^{j}M_{i}\times \sum_{j=1}^{k}{\left(k_{i}+k\right)}^{2}}. \end{array}$$

The statistical report of five different enterprise sales marketing oriented asset allocations is used for AI technology indicators under marketing based on the research findings. Based on statistics, the *HM*_*ij*_ represents the incident's approximate probability of occurring. The difference in coefficient is determined by responding to data about what potential benefits may be made and th decision is incorporate as given in equation (15) providing funding to such a marketing decision.

(14) $$\begin{array}{c} H=\sum_{i=1}^{j}\frac{M}{k}+\sum_{i=1}^{j}{\left(k_{i}+k\right)}^{2}+\int \frac{\sum H\times E\times h\times \sqrt{2\pi r}}{\sum M\times H_{ij}}. \end{array}$$

To investigate the correlation between marketing high level accounting talents and its benefits of purchasing from a specific supplier and the high level accounting talents benefits of purchasing from other distributors, use equation (15). Correlation testing is commonly used to assess such a correlation.

(15) $$\begin{array}{c} H\left(ME_{i}\right)=\sum_{i=1}^{j=1}\frac{M}{E}\times H_{i}^{\#}+\frac{M}{E}\times H_{i}^{*}+\sum_{i=1}^{j}{\left(k_{i}+k\right)}^{2}+\int \left(\frac{E}{2}+k_{j}\right)\times M\left(n|E_{i}=\;H_{ij}\right). \end{array}$$

## 3. Results and Discussion

Implementation of the unsupervised migration algorithm to analyze the employee or the new candidate's having high level accounting talent and also providing marketing oriented asset allocation is given in Figure 2. The tabulation of the graphical values is denoted in Table 1. The analysis is performed by considering the parameters such as marketing oriented asset allocation, high level accounting talents, training/testing, and accuracy. The domains where these combined talents were applied for analysis are marketing, engineer, consultant, sales, business, financial, and management. This novel model has resulted in better resultant percentage in the performance and a higher accuracy of 95.54% in the management application.

Next to the unsupervised migration algorithm analysis, online/offline marketing oriented asset allocation by the high level account talented candidate is represented in Figure 3. The application domain considered for the application is the same as that of the earlier analysis. But the candidate's performance in the online/offline marketing asset allocation is analyzed along with accounts talent and their maximum and minimum levels of marketing asset allocation are tabulated in Table 2. Similar to the earlier performance, management domain has obtained higher accuracy of 91.34% than any other domains.

Statistical online marketing analysis is presented in Figure 4. The analysis is carried out under market-oriented asset allocation, high level accounting talents, online statistical result marketing, and accuracy. In this analysis, the management domain obtained the best results compared to others. In addition to this, the sales have obtained 92.12% in marketing oriented asset allocation. In the other parameters, the proposed algorithms have shown increased accuracy and less fluctuation. The tabulation of this analysis is represented in Table 3.

In contrast to the above analysis, Figure 5 represents the statistical analysis in offline marketing mode. The values in the graph are tabulated in Table 4. From the results, it can be seen that the sales domain has provided higher performance results than the other domains.

The comparison analysis of the existing unsupervised migration algorithm based on deep learning with the existing Fractional Hausdorff Grey Model is depicted in Table 5. From the results, it can be observed that the proposed algorithm has obtained 99.12% accuracy, which is a 2.19% increase over the existing Fractional Hausdorff Grey Model.

## 4. Conclusions

High level accounting talent research asset allocation decisions are typically based on classification techniques used to categorize a set of measurements. An organization's overall marketing oriented asset allocation of high level accounting talents can be determined using historical data classification methods. This study used an unsupervised migration algorithm based on deep learning to analyze the performance of high level accounting talents. The results demonstrated that the proposed model outperformed the existing algorithms [30].

## Figures and Tables

**Figure 1:** Proposed model of AI in high level accounting.

**Figure 2:** Unsupervised migration algorithm using the marketing oriented asset allocation of high level accounting talents WSN with AI technology.

**Figure 3:** Performance analysis for online/offline marketing oriented asset allocation of high level accounting talents.

**Figure 4:** Analysis of statistical online marketing oriented asset allocation of high level accounting talents.

**Figure 5:** Analysis of statistical offline marketing oriented asset allocation of high level accounting talents.

**Table 1:** Result analysis unsupervised migration algorithm using the marketing oriented asset allocation of high level accounting talents WSN with AI technology.

Parameter	Marketing oriented asset allocation (%)	High level accounting talents (%)	Training/testing (%)	Accuracy (%)
Marketing	85.12	75.89	92.12	87.12
Engineer	82.34	80.12	90.24	84.72
Consultant	86.33	79.2	83.13	79.34
Sales	91.54	90.34	86.12	89.24
Business	95.23	94.32	91.56	93.87
Financial	89.12	92.12	85.23	86.90
Management	96.23	98.35	94.96	95.54

**Table 2:** The result analysis for online/offline marketing oriented asset allocation of high level accounting talents WSN with AI technology.

Parameter	Online/offline marketing oriented asset allocation (%)	High level accounting talents (%)	Minimum level marketing asset (%)	Maximum level of marketing asset (%)	Accuracy (%)
Marketing	84.83	94.23	64.23	70.23	86.67
Engineer	74.23	86.12	52.13	60.56	69.79
Consultant	72.12	75.12	57.35	65.35	65.23
Sales	90.12	92.88	69.3	95.65	89.31
Business	70.23	68.23	50.13	70.33	62.98
Financial	68.23	65.42	63.76	75.34	68.13
Management	92.12	94.23	85.78	95.99	91.34

**Table 3:** The result analysis of statistical online marketing oriented asset allocation of high level accounting talents.

Parameter	Marketing oriented asset allocation (%)	High level accounting talents (%)	Online statistical result marketing asset (%)	Accuracy (%)
Marketing	86.83	92.23	87.94	85.90
Engineer	77.23	84.12	82.45	82.89
Consultant	75.12	78.12	74.45	73.21
Sales	92.12	91.88	90.34	90.34
Business	77.23	66.23	73.56	75.83
Financial	65.23	69.42	66.87	64.23
Management	89.12	95.23	92.89	91.65

**Table 4:** Performance result analysis of statistical offline marketing oriented asset allocation of high level accounting talents.

Parameter	Marketing oriented asset allocation (%)	High level accounting talents (%)	Offline statistical result marketing asset (%)	Accuracy (%)
Marketing	89.68	93.74	89.49	86.19
Engineer	73.27	87.85	86.54	85.93
Consultant	78.64	75.92	78.46	77.54
Sales	94.78	94.34	92.43	91.47
Business	72.48	69.42	77.65	76.38
Financial	68.39	62.54	68.78	68.42
Management	90.73	91.38	89.98	90.46

**Table 5:** Comparison result for existing method marketing oriented asset allocation of high level accounting talents.

Algorithm	Online/offline marketing oriented asset allocation	Online/offline high level accounting talents	Statistical result (%)	Accuracy (%)
Unsupervised migration algorithm based on deep learning	92.45	98.23	95.72	99.12
Existing method: Fractional Hausdorff Grey Model	90.23	93.45	94.54	96.93

## Data Availability

The data used to support the findings of this study are available from the corresponding author upon request.
